# Bioinformatic Analysis and Cellular Assays Identify Substance P Influencing Th17/Treg Differentiation via the MyD88 Pathway as a Potential Contributor to the Progression of Asthma and Allergic Rhinitis

**DOI:** 10.1155/2022/3843954

**Published:** 2022-02-12

**Authors:** Yuemei Ma, Chang Liu, Guangpeng Xi, Yuanyuan Guan, Yao Tang, Jing Zhang, Yue Xu

**Affiliations:** ^1^Department of Allergy, The Second Affiliated Hospital of Harbin Medical University, China; ^2^Central Laboratory, Shenzhen Hospital of Beijing University of Chinese Medicine, China; ^3^Department of Allergy, The First Affiliated Hospital of Harbin Medical University, China

## Abstract

**Objective:**

This study is aimed at investigating the role of substance P (SP) in the development of asthma.

**Methods:**

The Gene Expression Omnibus (GEO) database was used to characterize SP expression in allergic rhinitis (AR) and asthma. Peripheral blood was collected from patients with asthma or AR. The expression of relevant cytokines and neuropeptides was measured. Enzyme-linked immunosorbent assay (ELISA) was also performed. The mast cell line LAD2 and the lung bronchial epithelial cell line BEAS-2B were treated with different concentrations of SP concentration. Then, the qRT-PCR method was used to determine the mRNA expression. Furthermore, p38 and p65 and their associated phosphorylated proteins (p-p38 and p-p65) were further validated by western blotting.

**Result:**

Clinical and GSE75011 data analysis suggested that MyD88 expression was upregulated in AR and asthma. Through the gene set variation analysis (GSVA), MyD88-related pathways were noticed and further investigated. ELISA results suggested that the SP expression was significantly increased in AR and asthma and IL-10 expression was decreased, whereas the expression of IL-6, IL-17A, IL-23, and TGF-*β* expressions increased. The mast cell line LAD2 was treated with different SP concentrations, and ELISA results showed that the expression of IL-6, IL-17A, IL-23, and TGF-*β* in the cell supernatant gradually increased with increasing SP concentrations, whereas that of IL-10 decreased. The lung bronchial epithelial cell line BEAS-2B was treated with different SP concentrations, and the expression of myeloid differentiation factor 88 (MyD88) and its related proteins was elevated. The expression of p38 and p-p38 proteins was elevated after SP treatment, and their expression levels elevated as SP concentrations increased. Finally, MyD88 expression at the single-cell level was also demonstrated.

**Conclusion:**

SP may affect the cytokine expression through the MyD88 pathway, thereby influencing Th17/Treg differentiation and eventually participating in the pathological process of asthma and AR. There are many pathological similarities between allergic rhinitis (AR) and bronchial asthma. In the present study, SP was found to possibly activate downstream inflammatory signaling pathways via MyD88, thereby affecting Th17/Treg differentiation and ultimately participating in the pathological process of asthma and AR.

## 1. Introduction

There are many pathological similarities between allergic rhinitis (AR) and bronchial asthma [1]. AR is an allergic reaction of the nasal mucosa triggered by an allergen, whose treatment is multimodal. In recent years, it has also been found to be associated with poor treatment outcome of deviated septum [1, 2]. Bronchial asthma (hereinafter referred to as asthma) is a chronic airway inflammatory disease [3]. Both diseases occur in allergic and pediatric populations, and although AR is generally mild, some studies suggest that AR has a high potential to trigger bronchial asthma [4]. Epidemiological studies have shown a strong association between bronchial asthma and AR, with a high overlap in the disease distribution of bronchial asthma and AR [5]. Overall, the prevalence and burden of AR and asthma are particularly high, ranging between 1% and 20% [6]. Currently, approximately 300 million patients have been diagnosed with asthma worldwide, and the incidence rate is approximately 13-20% [7]. This means that the search for comorbid mechanisms of AR and asthma has significant clinical implications.

Pathogenesis of AR and asthma has not yet been completely elucidated owing to the complex influence of environmental and genetic factors, such as immune-inflammatory response, neural, and airway hyperresponsiveness mechanisms [8, 9]. Inflammation associated with asthma and AR is thought to be mediated by the involvement of multiple cells and cytokines. Cellular interactions play an important role in the development of disease [9–11]. Phenotypic induction of regulatory T cells (Tregs) is a hallmark of successful allergen immunotherapy [12]. There are two types of Treg cells: natural regulatory T lymphocytes, which exert regulatory effects mainly in a cell-to-cell contact signaling manner, and adaptive regulatory T lymphocytes (iTreg), including type I regulatory T cells (Tr1) and Th3 cells, which mainly downregulate immune responses by secreting interleukins (IL-10) and transforming growth factor-*beta* (TGF-*β*) [13]. Th17 and Treg cells are derived from a common initial T cell population with differentiation shifted by different environments to maintain immune homeostasis by suppressing and balancing each other's differentiation functions [14]. Recent studies have shown that the balanced relationship between Th17 and Treg cells may play an important role in the development of allergic asthma and AR [15, 16]. Doganci et al. reported that decreased Treg-cell level in an asthma mouse model can lead to enhanced airway hyperresponsiveness [17].

Various neuropeptides, such as substance P (SP), are widely present in the blood and are closely associated with respiratory inflammation, T-helper cell balance, and mucus secretion [18, 19]. SP plays a key role in this process [20]. Therefore, dysregulation of balance between T lymphocytes and cytokines is important in the development of asthma as well as AR. However, studies investigating the association between SP expression and Th17/Treg cells were very limited.

In this study, different concentrations of SP were used to treat mast cell line LAD2 and bronchial epithelial cell line BEAS-2B to explore the effect of SP on asthma, thus providing a theoretical basis for clinical diagnosis and treatment. We aimed to investigate the role of substance P (SP) in the development of asthma.

## 2. Materials and Methods

### 2.1. Bioinformatic Data Acquisition and Analysis

The GSE75011 dataset from the GEO (http://www.ncbi.nlm.nih.gov/geo/) database was used for this study, which included 40 asthma patients, 25 AR patients, and 15 normal individuals [21]. Transcriptome analysis of T cells in circulating blood from the GSE75011 dataset revealed that asthma and AR share common sensitizing factors. Gene set variation analysis (GSVA) was used to quantify the expression of pathways in each sample, completed by using the “GSVA” R package [22–24]. Single cells play an important role in revealing the heterogeneity of tissue and gene expression [25, 26]. Single-cell expression profile data of MyD88 in bronchial cells were obtained from Tabula Muris (https://tabula-muris.ds.czbiohub.org/), a single-cell transcriptome profile for Mus mucus [27–29].

### 2.2. Blood Samples

Human blood specimens were obtained from patients and normal controls, and all blood samples were collected and rapidly centrifuged to collect the serum, and samples were stored in an ultralow temperature refrigerator at 80°C. All samples were collected following the ethical guidelines of The Second Affiliated Hospital of Harbin Medical University, and all study participants signed informed consent.

### 2.3. Cells and Cell Culture

The normal bronchial epithelial cells BEAS-2B and human mast cell line LAD2 were purchased from the Institute of Chinese Academy of Sciences, Shanghai, China, where BEAS2B was cultured with the BEGM medium in a 5% CO_2_ incubator at a constant temperature of 37°C, and LAD2 cells were cultured in high-glucose Dulbecco's Modified Eagle's Medium supplemented with 10% foetal bovine serum (FBS) and 1% double antibodies.

### 2.4. RNA Extraction and qRT-PCR

RNA was extracted from blood samples and cells using TRIzol based on the TRIzol procedure; subsequently, RNA was reverse transcribed to cDNA using the Promega Reverse Transcription Kit. cDNA was quantified using TB Green premixed PCR reagent to monitor mRNA levels. Relative mRNA levels were calculated using the 2-*ΔΔ*Ct method and using the glyceraldehyde 3-phosphate dehydrogenase (GAPDH) as an internal reference.

### 2.5. Protein Extraction and Western Blotting

BEAS-2 cells were treated with SP-1 (0.5, 1, and 2 *μ*mol/L), and protein extraction was performed after 24 h. RIPA (Beyotime) plus protease and phosphatase were used. Equal amounts of proteins were subjected to gel electrophoresis using 10% sodium dodecyl sulphate–polyacrylamide gel (Yamei) at a constant voltage of 120 V for 100 min; the gel was transferred onto polyvinylidene difluoride membranes at a constant flow of 300 mA for about 60–90 min, followed by room temperature closure treatment with 5% BSA for 1 h and incubation with primary antibody overnight. On the next day, the proteins were treated with the corresponding secondary antibody for 2 h at room temperature, and the collection was performed on a developer (Tanon). Primary antibodies included anti-GAPDH (CST), anti-p38 (CST), anti-p-p38 (CST), anti-p65 (CST), and anti-p-p65 (CST), and GAPDH was used as an internal reference.

### 2.6. Enzyme-Linked Immunosorbent Assay (ELISA) for Serum and Cell Supernatant

Human sera were diluted 100-fold, and the expression of IL-6, IL-10, IL-17A, IL-23, TGF-*β*, and SP-1 was determined via ELISA using the Invitrogen ELISA kit according to the manufacturer's instructions. LAD2 cells were treated with SP-1 (0.5, 1, and 2 *μ*mol/L) for 24 h, and supernatants were collected and assayed using the Invitrogen ELISA kit.

### 2.7. Statistical Methods

All experiments were performed at least thrice. All data were presented as mean ± standard deviation. The chi-squared test was used for statistical analysis of frequencies between two groups, *t*-test was used for statistical differences between two independent samples, and *p* value ≤ 0.05 was considered statistically significant.

## 3. Results

### 3.1. SP Expression Was Elevated in Patients with Asthma

To determine the neuropeptide expression in patients with asthma, the peripheral blood of patients with asthma was tested using qRT-PCR for the expression of relevant neuropeptides, including SP, neurokinin A (NKA), NKB, calcitonin gene-related peptide (CGRP), vasoactive intestinal polypeptide (VIP), gamma-aminobutyric acid (GABA), and neuropeptide Y (NPY). The expression of SP, CGRP, and VIP was found to be higher than that in asthmatic patients, with a more pronounced increase in SP expression (Figure 1(a)). Therefore, SP in the serum was measured via ELISA, and a significant increase in SP expression was found in patients with AR (Figure 1(b)). Based on the GSE75011 dataset, MyD88 was also found to be highly expressed in AR patients (Figure 1(c)). The activity of the MyD88-independent TLR4 cascade pathway was quantified and ranked (from 1 to 80) for each sample in GSE75011 by GSVA. The MyD88-independent TLR4 cascade pathway was found to be activated in asthmatics and AR patients (Figure 1(d)).

### 3.2. Proinflammatory Factors Were Elevated in Patients with Asthma

Immunity plays an important role in asthma and AR, including abnormalities in the adaptive and humoral immunity and Th1/Th2 and Th17/Treg imbalance [30–32]. To determine the cytokine profile in patients with asthma, cytokine expressions, including IL-2, IL-4, IL-6, IL-10, IL-17A, IL-23, and TGF-*β*, in the peripheral blood cells of patients with asthma were measured, and it was found that the expression of IL-6, IL-17A, IL-23, and TGF-*β* was elevated, whereas that of IL-2 and IL-10 was decreased (Figure 2(a)). To further determine the cytokine profile, IL-6, IL-10, IL-17A, IL-23, and TGF-*β* were also measured using ELISA, and it was found that the expression of IL-10 was decreased, whereas that of IL-6, IL-17A, IL-23, and TGF-*β* was higher than that in normal participants (Figure 2(b)). In conclusion, SP was speculated to influence cytokine release, affecting the pathogenesis of asthma.

### 3.3. SP Promoted the Expression of Mast Cell Proinflammatory Factor

Previous studies have reported the involvement of mast cells in the pathogenesis of asthma [33]. Therefore, we treated the mast cell line LAD2 with different SP concentrations and assessed the expression of IL-6, IL-10, IL-17A, IL-23, and TGF-*β* cytokines using ELISA to investigate the inflammatory mechanism of SP on asthma. The results showed that the expression of IL-6, IL-17A, IL-23, and TGF-*β* in the cell supernatant gradually increased with increased SP concentration, whereas that of IL-10 was decreased (Figure 3). Previous studies have reported that IL-6 and TGF-*β* are closely associated with the differentiation of Th17 [34], IL-10 is closely related to Treg [35], and Th17/Treg is involved in the mechanism of asthma [31]. In conclusion, SP may influence the mechanism of asthma development through Th17/Treg.

### 3.4. SP May Be Involved in the Mechanism of Asthma through the Myeloid Differentiation Factor 88 (MyD88) Pathway

A previous study reported that SP affected cytokine changes in asthma; however, the specific mechanism remains unclear. Some studies have found that SP can affect the IL-6 and TNF-*α* expression in mast cells through the NF-*κ*B pathway [36], whereas NF-*κ*B is also involved in the SP mechanism on asthma [37]. Another study found that SP can be involved in disease development through the MyD88 pathway [38]. Therefore, the lung bronchial epithelial cell line BEAS-2B was treated with different SP concentrations. First, RT-PCR was used to determine the mRNA expression, and it was found that the expression of MyD88 and its related proteins IRK4, TRAF6, and MKK3 was elevated. In addition, the expression of the NF-*κ*B pathway protein NFKB1 was elevated but was not significant (Figure 4(a)). To further verify the results, western blotting was used to detect p38 and p65 and their related phosphorylated proteins (p-p38 and p-p65), which revealed no significant changes in the expression of p65 and p-p65 in SP-treated cells (Figure 4(b)). These results suggested that NF-*κ*B was not involved in the regulation of cytokine expression in asthma despite SP treatment. Further analysis revealed that the expression of p38 and p-p38 was elevated after SP treatment, and their expression levels increased with the increasing SP concentration (Figure 4(c)), which concluded that SP may affect the cytokine expression through the MyD88 pathway but not through the NF-*κ*B pathway. In addition, correlation analysis showed that the MyD88-independent TLR4 cascade pathway was significantly and positively correlated with MyD88, NFKBIA, IKBKB, NFKB1, TAB1, IRAK1, IRAK4, and TRAF6 (Figure 4(d)). The single-cell profile of Tabula Muris showed that MyD88 was widely expressed in bronchial cells (Figure 4(e)).

## 4. Discussion

The classical pathogenesis of asthma as well as AR is thought to be an inflammatory response triggered by the interaction of cells and cell-signaling molecules [39]. However, a majority of atopic patients do not develop asthma in the presence of sustained allergen exposure, suggesting that additional mechanisms act in concert with type 2 immunity to facilitate the pathogenesis of asthma; however, these additional mechanisms have not yet been comprehensively elucidated. Our study shows that SP may activate downstream inflammatory signaling pathways through MyD88, thereby affecting Th17/Treg differentiation and ultimately participating in the pathological process of asthma and AR.

SP was found to be increased in the sputum and alveolar lavage fluid of patients with asthma [40, 41] and in nasal secretions of patients with AR [42]. It can also cause many typical changes in the airways of patients with asthma [43], including bronchoconstriction, increased mucus secretion, and plasma leakage [44]. SP mainly acts through the neurokinin 1 receptor (NK1R) [45]. Studies have shown that NK1R expression is upregulated in the lungs of patients with asthma compared to healthy controls [46]. NK1R expression on the mast cells is thought to be functionally relevant and results in increased sensitivity of the mast cell [47]. Furthermore, studies with functional analyses have suggested that SP stimulates inflammation by increasing TNF-*α* production in mouse mast cell lines and that these effects are dependent on NK1R [47]. Mast cells originate from the CD34+ CD117+ bone marrow pluripotent hematopoietic progenitor cells, with precursor cells that enter the circulation in an immature state and complete their tissue-specific differentiation and maturation in specific peripheral tissues [48]. Mast cells are widely distributed in tissues and are mainly present at the contact surfaces between the host and external environment, such as the skin, respiratory mucosa, and epithelial tissues of the gastrointestinal tract. Mast cell degranulation plays a key role in allergic diseases [49, 50]. The presence or accumulation of mast cells in certain compartments of the lungs is a pathological characteristic of allergic asthma [51]. Patients with asthma have an increased number of mast cells in their airway smooth muscles. The number of mast cells in the smooth muscles was also higher in patients with allergic asthma than those with nonallergic asthma. In this study, SP expression was found to be significantly increased in patients with asthma, and the concentration of IL-6, IL-17A, IL-23, and TGF-*β* in the supernatant of the mast cell line LAD2 gradually increases as the SP concentration increased, whereas that of IL-10 decreased. This finding suggests that SP acts on NK1R in the surface of mast cells to increase the secretion of IL-6, IL-23, and TGF-*β* by the mast cells, whereas IL-10 secretion is decreased.

SP has been shown to regulate the messenger RNAs (mRNAs) of toll-like receptors (TLRs) in human mast cells [52]. It can also upregulate TLR4 expression. Some allergens can stimulate TLRs, which may play a role in asthma development. TLRs could induce various inflammatory factors upon activation, such as TNF-*α*, IL-1*β*, and IL-6, which play an important role in the inflammatory process of acute gout [53–55]. The TLR4 expression in human lung mast cells has also been confirmed [56]. *In vivo*, TLR4-mediated mast cell activation was reported to enhance the mast-cell-deficient allergic airway inflammatory cell model and cytokine release [57]. MyD88 is a key junction molecule in the TLR signaling pathway and plays an important role in the transmission of upstream information and disease development. In this study, the expression of MyD88 and its related proteins IRK4, TRAF6, and MKK3 was elevated in the lung bronchial epithelial cell line BEAS-2B treated with different SP concentrations, and that of the NF-*κ*B pathway protein NFKB1 was also elevated; however, NF-*κ*B elevation was not significant; further western blot detection revealed that the expression of p65 and p-p65 did not significantly change; the expression levels of p38 and p-p38 were elevated and increased as the SP concentration increased. Therefore, SP may affect cytokine expression through the MyD88 pathway, while NF-*κ*B, one of the downstream transcription factors of MyD88, may not be activated in significant amounts.

IL-10 and IL-6 also play an important role in mediating Th17/Treg differentiation. IL-10-secreting Treg cells suppress the Th2-type immune response (IL-4, IL-5, and IL-13) and IL-17-secreting Th cells [58–60]. IL-10 plays an important role as a regulatory molecule in the innate and adaptive immune responses, which commonly leads to immune tolerance or suppression of human tissue inflammation. Immune tolerance is usually directed against any immune-activating molecules and several immune mechanistic mediators [61]. Once the immune tolerance fails, the overwhelming immune effects and inflammatory functions frequently result in allergies, asthma, neoplasms, chronic infections, transplant rejection, graft-versus-host disease, and other autoimmune diseases [62, 63]. IL-6, a pleiotropic factor, is one of the important cytokines involved in immune regulation and inflammatory responses. IL-6 is considered a central regulator of immune and inflammatory processes. IL-6 induces Th17 differentiation with TGF-*β* [64, 65]. TGF-*β* is required for Th17 and Treg differentiation and induces Foxp3 expressions [66]. IL-6 acts as an effective proinflammatory cytokine in T cells by promoting Th17 differentiation and inhibiting Treg differentiation, suggesting that controlling IL-6 normalises the balance between Th17 and Treg cells and may alleviate autoimmune symptoms [34]. The low numbers of natural Treg cells (nTregs) at birth are associated with subsequent food allergies. The balance between Th17 and Treg is essential for immunity-specific homeostasis.

From this study, we can define that high SP expression of asthma and AR leads to the upregulation of TLR of mast cell membrane by binding to the NY1R on mast cell surface, increased secretion of IL-6, IL-23, and TGF-*β*, and decreased secretion of IL-10 in response to allergen stimulation. MyD88 plays a key role of message transduction. The gene set variation analysis (GSVA) score analysis also showed that activation of the MyD88 pathway is closely associated with allergic diseases. And then, high expression of IL-6, IL-23, and TGF-*β* promotes Th17 differentiation together, disrupting the Th17/Treg balance and elevating IL-17 expression, leading to the development of asthma. However, the beneficial effects of histamine receptor antagonists are limited owing to several mediators secreted by the mast cells. Patients with allergic asthma cannot be effectively treated by targeting another single mast-cell mediator. Therefore, other triggers of mast cell activation, which may contribute to the occurrence of different symptoms in patients with allergic asthma, should be identified to develop new mast cell-targeting drugs. In addition, the transcriptomic data of the GSE75011 dataset were derived from Th2 cells, which were biased from the Th17/Treg balance involved in this study, but still showed certain reference significance.

## 5. Conclusion

Allergic rhinitis (AR) shares many pathological similarities with bronchial asthma. In this study, we used bioinformatics and cellular experiments to discover that SP may activate downstream inflammatory signaling pathways through MyD88, thereby affecting Th17/Treg differentiation and ultimately participating in the pathological process of asthma and AR. However, further animal experiments and more in-depth studies are needed.

## Figures and Tables

**Figure 1:** SP expression was elevated in patients with asthma and AR. (a) The RT-PCR results showing the elevated expression of SP, CGRP, and VIP in patients with asthma. (b) The ELISA results showing the elevated expression of SP in patients with asthma. (c) The expression characteristics of MYD88 in the GSE75011 dataset. (d) The activity of the MYD88-independent TLR4 cascade pathway was quantified and ranked from 1 to 80 for each sample in GSE75011 by GSVA. MyD88-independent TLR4 cascade pathway found to be activated in asthma and AR patients (^∗^*p* ≤ 0.05 and ^∗∗∗^*p* ≤ 0.001).

**Figure 2:** Elevated expression of proinflammatory factors in (a) asthma and (b) AR.

**Figure 3:** SP promotes the secretion of mast cell proinflammatory factors. With increasing SP concentrations, the concentration of (a) IL-6, (b) IL-17A, (c) IL-23, and (d) TGF-*β* increased and the concentration of (e) IL-10 decreased in the supernatant of LAD2 cells (^∗^*p* ≤ 0.05, ^∗∗^*p* ≤ 0.01, and ^∗∗∗^*p* ≤ 0.001).

**Figure 4:** SP can activate MyD88 pathway. (a) qRT-PCR results showing that MyD88, IRAK4, TRAF6, MKK3, and NFKB1 genes were upregulated in BEAS-2B cells after SP (1 *μ*mol/L) treatment. (b) No significant difference in the expression of p65 and p-p65 is observed in BEAS-2B cells after SP treatment. (c) Protein expression of p38 and p-p38 is elevated after SP treatment. (d) Correlation analysis of MyD88-independent TLR4 cascade pathway and MYD88, NFKBIA, IKBKB, NFKB1, TAB1, IRAK1, IRAK4, and TRAF6. (e) Characterization of the MyD88 expression in bronchial cells. ^∗^*p* ≤ 0.05 and ^∗∗^*p* ≤ 0.01.

## Data Availability

The GSE75011 dataset from the GEO database was used for this study. Single-cell expression profile data of MyD88 in bronchial cells were obtained from Tabula Muris (https://tabula-muris.ds.czbiohub.org/). Clinical data can be obtained by contacting the corresponding author with a reasonable request.

## Abbreviations

CGRP: Calcitonin-gene-related peptide
GABA: Gamma-amino butyric acid
Tregs: Adaptive regulatory T lymphocytes
NKA: Neurokinin A
NK1R: Neurokinin 1 receptor
NPY: Neuropeptide Y
nTregs: Natural Treg cells
SP: Substance P
TGF-*β*: Transforming growing factor-*β*
TLRs: T toll-like receptors
Treg cells: Regulatory T cells
Tr1: Type I regulatory T cells
VIP: Vasoactive intestinal polypeptide.
